This article has been retracted.

# Facial Mask Detection Using Depthwise Separable Convolutional Neural Network Model During COVID-19 Pandemic

**DOI:** 10.3389/fpubh.2022.855254

**Published:** 2022-03-07

**Authors:** Muhammad Zubair Asghar, Fahad R. Albogamy, Mabrook S. Al-Rakhami, Junaid Asghar, Mohd Khairil Rahmat, Muhammad Mansoor Alam, Adidah Lajis, Haidawati Mohamad Nasir

**Affiliations:** ^1^Center for Research & Innovation, CoRI, Universiti Kuala Lumpur, Kuala Lumpur, Malaysia; ^2^Institute of Computing and Information Technology, Gomal University, Dera Ismail Khan, Pakistan; ^3^Computer Sciences Program, Turabah University College, Taif University, Taif, Saudi Arabia; ^4^Research Chair of Pervasive and Mobile Computing, Information Systems Department, College of Computer and Information Sciences, King Saud University, Riyadh, Saudi Arabia; ^5^Faculty of Pharmacy, Gomal University, Dera Ismail Khan, Pakistan; ^6^Faculty of Computing, Riphah International University, Islamabad, Pakistan; ^7^Malaysian Institute of Information Technology, University of Kuala Lumpur, Kuala Lumpur, Malaysia; ^8^Faculty of Computing and Informatics, Multimedia University, Cyberjaya, Malaysia; ^9^Faculty of Engineering and Information Technology, School of Computer Science, University of Technology Sydney, Ultimo, NSW, Australia

**Keywords:** facial image classification, Depthwise Separable Convolutions, face mask detection, deep learning, MobileNet

## Abstract

Deep neural networks have made tremendous strides in the categorization of facial photos in the last several years. Due to the complexity of features, the enormous size of the picture/frame, and the severe inhomogeneity of image data, efficient face image classification using deep convolutional neural networks remains a challenge. Therefore, as data volumes continue to grow, the effective categorization of face photos in a mobile context utilizing advanced deep learning techniques is becoming increasingly important. In the recent past, some Deep Learning (DL) approaches for learning to identify face images have been designed; many of them use convolutional neural networks (CNNs). To address the problem of face mask recognition in facial images, we propose to use a Depthwise Separable Convolution Neural Network based on MobileNet (DWS-based MobileNet). The proposed network utilizes depth-wise separable convolution layers instead of 2D convolution layers. With limited datasets, the DWS-based MobileNet performs exceptionally well. DWS-based MobileNet decreases the number of trainable parameters while enhancing learning performance by adopting a lightweight network. Our technique outperformed the existing state of the art when tested on benchmark datasets. When compared to Full Convolution MobileNet and baseline methods, the results of this study reveal that adopting Depthwise Separable Convolution-based MobileNet significantly improves performance (Acc. = 93.14, Pre. = 92, recall = 92, *F*-score = 92).

## Introduction

Prior to the coronavirus disease 2019 (covid-19) pandemic, there was no concrete evidence supporting the use of community masks to reduce the spread of respiratory infections. Masks are primarily intended to prevent the wearer from spreading the viral droplets (source control). Covid-19 and other respiratory infections spread primarily through inhalation of respiratory aerosols produced by coughing, sneezing, talking, or breathing. The virus propagates and migrates down the respiratory tract and may lead to pneumonia, acute respiratory distress syndrome (ARDS) and even death. The ongoing pandemic and the rapidly emerging variants have made this respiratory illness, a daily headline. To prevent the spread of infection, it is recommended that people use face masks as part of their personal safety gear and as a public health measure (1, 2). In light of this, the development of a system that can identify people wearing masks is critical in today's world.

Scientists have attempted to build automated facial mask recognition systems in public locations to ensure the use of face masks in common areas. Following the COVID-19 epidemic, other researchers developed their own techniques for monitoring face masks in common areas. Employing image processing algorithms, Surveillance systems are utilized for monitoring of public spaces in order to guarantee that no one's face is visible in crowded locations (2). Deep learning-based approaches for object identification and imagery analytics have been increasingly popular over the years. The majority of the past research has been conducted using convolutional neural network models. There are two instances in which current face mask detection algorithms are unable to reliably identify the masks. When there is a large number of people in a single image or video frame, it is difficult to precisely identify all of the faces “with mask and without mask.” In our nation, ladies wear half-faced veils that serve the same purpose as face masks, but the current methods do not identify them as face masks.

How to construct a more efficient and accurate classification approach is a key aspect for the implementation of facial mask detection techniques in mobile environment. However, several deep learning models are costly and time-consuming in their evaluation steps, making them unsuitable for mask detection in the facial image paradigm in a mobile environment. In order to overcome the shortcomings of the existing approach, the suggested method makes use of Depthwise Separable Convolutions with MobileNet for mask detection in facial images (3). Depthwise separable convolution (DSC) was first proposed in (4) and is now widely used in image processing for classification tasks (5).

### Research Motivation

There has been a tremendous amount of interest in deep learning in the past few years, notably in fields like machine vision, text analytics, object recognition, and other information processing aspects (6). The majority of the past research in object detection has been conducted using convolutional neural network models. Using deep learning architectures, convolutional neural networks (CNNs) have become more popular in recent years for a variety of tasks, such as picture identification (2), speech synthesis (7), object tracking (8), and image thresholding (9). When it comes to the abovementioned domains, CNN exhibits an excellent capacity to retrieve features from images. A growing number of research methods are replacing traditional classification methods with CNNs in order to more effectively capture image information and achieve improved classification performance. Due to energy limitations, numerous deep neural networks are unsuited for mobile-based facial image classification since their evaluation phase is time consuming and expensive. We describe a MobileNet-based facial image classification model that uses a Depthwise separable convolution technique to handle this problem (2). DSC (Depthwise separable convolution) was first presented in (4) and is commonly used in image processing for classification tasks (10). The Depthwise separable convolution is a quantized version of the ordinary convolution. Convolutions are often separated into Depthwise and 1×1 pointwise convolutions. Rather than applying each filter to all input channels as in traditional convolution, the Depthwise convolution layer applies one filtering to one pulse and then uses a 1×1 pointwise convolution to combine the Depthwise convolution results. Depthwise separable convolution reduces the number of learnable parameters and the expense of test and train computations.

### Problem Statement

COVID-19 is a highly contagious disease, and the WHO and other health agencies have recommended that people use face masks to prevent its transmission. All governments are attempting to guarantee that face masks are worn in public places, but it is difficult to manually identify those who are not wearing face masks in crowded places. Scientists are working on developing automatic methods to identify and enforce the use of face masks in public locations. The problem may be summarized as follows: given a face picture as an input, the classification model must categorize the facial image in a mask detection task using the classification model. Using Depthwise Separable Convolutions with MobileNet data, we provide a method for mask detection-driven face picture classification that is both fast and accurate, as demonstrated in this work. We employed Depthwise separable convolution layers instead of traditional convolutional layers to successfully develop the model with a smaller number of learnable parameters and a smaller number of learnable parameters.

### Research Questions

In this study, a Depthwise Separable Convolution Neural Network (DS-CNN) technique based on MobileNet is used to achieve rapid and accurate classification results utilizing the Softmax function. The goal of this study is to identify face masks from facial photographs.

The research questions proposed in the paper are listed in Table 1.

**Table 1:** Investigative research questions.

**Research question**	**Motivation**
RQ1. How can the Depthwise Separable Convolutional Neural Network based on MobileNet be utilized to successfully categorize photos for facial mask detection?	Investigate the Depthwise Separable Convolution Neural Network based on MobileNet to learn how it may be used to classify facial photos for mask recognition.
RQ2. How efficient is the suggested technique in contrast to the traditional CNN model in terms of many performance assessment measures?	Examine the usefulness of the proposed deep learning model, MobileNet-based Depthwise Separable Convolution Neural Network, which classifies face photos in terms of mask recognition using a variety of performance metrics such as accuracy, recall, F1 measure, and precision.
RQ3 What is the effectiveness of the suggested approach in comparison to comparable approaches?	Compare the efficacy of the proposed mobile-based deep learning model employing depth-wise separable convolution in categorizing face pictures to baseline testing using a variety of assessment measures including precision, recall, F1-score, and accuracy.

### Research Contributions

The following is a list of the study's most significant contributions:

- We describe an effective face mask-based facial image classification system using a MobileNet-based deep learning model with a Depthwise separable convolution approach.
- Faster training with fewer parameters is possible with the proposed multilayer MobileNet-based model.
- With Depthwise separable convolution units, we synthesize mobile-based input patterns (facial pictures) using their internal memory layouts and resource consumption.
- To combat overfitting, we employ a dropout strategy in which neurons are switched off at random times during training.
- When evaluated on a publicly accessible dataset, the suggested strategy outperforms current state-of-the-art image classification methods.
- Based on publicly accessible datasets for the identification of face masks, we compared our suggested technique to a baseline study on the same dataset.

The following is a breakdown of the article's structure: Following the evaluation of similar studies in part 2, section Methodology, focuses on methodology, and section Results and Discussion provides findings and analysis. Conclusions and future prospects are discussed in section Conclusion and Future Work.

## Related Work

Face mask detection is a subset of object recognition that uses image processing algorithms. Digital image processing may be divided into two broad categories: classical image processing and deep learning-based image analysis. As opposed to classical image analysis, which uses complex formulas to recognize and interpret pictures, deep learning-based approaches utilize models that mimic the workings of the human brain. Deep Learning models have been used in the majority of past research. After correctly recognizing the face in the picture or video, the CNN-based approach by Kaur et al. (2) evaluates if the face has been disguised. It is also capable of identifying a moving face and a mask in a video as a surveillance job performance. Accuracy is great with this method. An algorithm called YOLO-v3 was developed by Bhuiyan et al. (11) to identify face masks in public spaces. They trained the YOLO-v3 model on their own custom dataset of photos with people labeled as “mask and no-mask.” The model's performance was enhanced by Mata (12) via data augmentation. It is necessary to create a CNN model that can distinguish between ROIs with and those without a face mask in order to extract the facial area as a ROI. With the use of Mobile NetV2, Toppo et al. (1) developed a method for detecting face masks that incorporates three distinct face detector models in order to test the model's correctness and evaluate its performance. The trained model's outcome allows for implementation on low-power devices, making the mask detection method's inclusion faster than previous strategies. To recognize people who were not wearing face masks in government workplaces, Balaji et al. (13) utilized a VGG-16 CNN model developed in Keras/TensorFlow and Open-CV to detect people who were not wearing face masks. To compensate for the model's light weight, Fan et al. (3) offered two additional methods. A unique residual contextual awareness module for crucial face mask regions Two-stage synthetic Gaussian heat map regression is used to identify better mask discrimination features. Ablation research has found that these strategies can improve feature engineering and, as a result, the effectiveness of numeric identification. For AIZOO and Moxa3K, the suggested model outperforms prior models.

Conventional deep learning algorithms for lightweight facial image classification alone do not give a good discriminating feature space, as shown by the research covered above, and they complicate the model and greatly increase the number of parameters and necessary computational resources.

In this study, a Depthwise Separable Convolution Neural Network-based MobileNet for the detection of face masks by classifying facial images is developed in this study in an effort to answer the shortfalls of previous research in this area (2). Our technique improves the work performed by (2) by replacing the conventional convolution with a depth-wise separable convolution in the neural network (14). Table 2 shows a tabular summary of selected earlier works.

**Table 2:** A partial list of literature review works.

**Study**	**Technique**	**Results**	**Limitations**
Toppo et al. (1)	Mobile NetV2	88%	Revised parameter settings can improve the system performance
Kaur et al. (2)	CNN-based approach	86%	Light weight DWS-based CNN can provide more efficient results
Fan et al. (3)	Residual contextual awareness module	91% (Acc.)	Due to the constraints of the datasets, more processing is necessary to generate visualizations.
Bhuiyan et al. (11)	YOLO-v3 model	86% (Acc)	YOLOv4 needs to be compared using the proposed model.
Mata (12)	CNN model	60 % (Acc)	More effective techniques required for improved results
Balaji et al. (13)	VGG-16 CNN	N/A	DWS solution can provide better results

### Research Gap

Several machine and deep learning models, however, are costly and time-consuming in their evaluation phase due to energy restrictions, making them unsuitable for facial image categorization in terms of mask detection. We propose a depth-separable convolutional neural network based on MobileNet for facial image classification to tackle the issue of mask detection. The proposed strategy, which involves optimizing the system configuration and specifications, has the potential to satisfy the needs of real-time applications while maintaining a high level of accuracy.

## Methodology

The major phases in our suggested technique are illustrated in Figure 1.

**Figure 1:** Generic Diagram of proposed system.

### Overview of the Proposed System

The following is a quick summary of the suggested approach.

***Dataset Collection:*** Images from various sources are used to build a dataset. The size of datasets can be expanded by the application of data enhancement techniques. The photographs are stored in two files, “training dataset” and “test dataset,” each of which comprises 80 and 20% of the images, respectively. Bounding boxes, sometimes known as “data annotations,” are created around an area of interest using a variety of methods. Labeling pictures as “mask” or “NO mask” will be done using the LabelImg tool in the proposed system.

***Image Enhancement***: To draw attention to the foreground elements, the image is improved through preprocessing methods and segmentation techniques.

***Model Implementation***: We ran the tests on an Intel Core i7 processor with an Nvidia GTX 1,080 graphics card and Windows 10. Python 3.5 was used as the programming language in this project.

***Training the model:*** To distinguish between those wearing “masks” and those who aren't, the model is trained in an online GPU environment called Google Colab. A folder referred to as “the trained folder” is used for training purposes.

***Prediction***: Using the test folder, the model is tested for its ability to identify and classify masks and no-masks that were found in the original photos.

### A Detailed Overview of the Proposed System

This section describes the research approach (Figure 2). The fundamental purpose of our method is to provide a depth-wise separable convolution-driven MobileNet solution for mask or no-mask detection in facial image classification. The system receives source data from a variety of datasets as input, and the outcome is the categorization of the input face image into two categories, namely, mask and no-mask data. The dataset utilized and the proposed approach are detailed in the following subsections:

**Figure 2:** Proposed Framework with detailed view.

#### Data Collection

All phases of image analysis research necessitate the use of data, from training algorithms to assessing their performance. The following datasets were employed in this study:

1. **Dataset for Identification of Aizoo Face Masks**

A fully accessible dataset called AIZOO face mask identification was generated by AIZOOTech (15) by integrating roughly 8,000 photos from the WIDER FACE (16) and MAsked FAces (MAFA) (17) datasets and re-annotating them to meet the face mask recognition scenario. A reasonable balance was achieved when Wider Face (50%) contributed the majority of regular faces and MAFA (50%) contributed the majority of mask-wearing faces, ensuring a reasonable balance between the two. For the purposes of testing, just a sample of 1,839 photographs had been selected (18).

2. **Face Mask Identification Data source by Moxa3K**

Face mask investigations may be made easier with the Moxa3K facial masking identification dataset (19). It has 3,000 photos, 2,800 of which are for training and 200 for testing. In order to build the dataset, Kaggle photos and pictures from the Web were combined. A downside of the database is that it only comprises small face images that are not covered by masks.

***Train/Test Subsets**:* In order to develop a CNN model, you need a large amount of data. As the number of photos in the dataset grows, so does the model's accuracy. A training dataset and a test dataset each comprise 80 and 20% of the photos, respectively. A sample listing is shown in Figure 3.

**Figure 3:** **(A,B)** A sample dataset of mask and no-mask images.

#### Preprocessing

Preprocessing methods and picture segmentation are used to improve the input image in order to draw attention to the foreground items. For this, we preprocess all of the photographs in the folders and adjust the height and width dimensions to 224 × 224, respectively, to make our data more consistent and also because it is the dimension recognized by MobileNet. The photos were saved in an array format from the “Keras.preprocessing.image” module, which is necessary while using MobileNet designs. One-hot encoding was accomplished by utilizing LabelBinarizer for the attributes (tags) “mask” and “no-mask,” which were needed while using MobileNet models (20).

***Image Labeling***: Dataset labeling is a process that involves drawing rectangles over a region of investigation using a range of tools. The LabelImg tool (21) is used in the proposed system to identify the pictures as “Mask” or “NO Mask,” depending on their content. Figure 4 depicts the preprocessing used for the final cut (22).

**Figure 4:** Preprocessing by drawing rectangles.

#### Classic vs. Depthwise Separable Convolutions

This work makes use of a Depthwise Separable Convolutional Neural Network based on MobileNet for classification. To construct the Depthwise Separable Convolutional Neural Network based on MobileNet, we'll go over the techniques employed in this part. Depthwise separable convolutions are being proposed to replace the currently expensive convolutional layers used in image recognition software. Weights and calculation time are both reduced using Depthwise separable convolution. There is an overview of the formulas and fundamental components of the approaches, followed by a detailed description of the proposed approach for effective classification of face photos in the COVID-19 scenario.

#### Classic Convolution

In deep learning, the traditional convolution is often referred as the standard or classic convolution. Figure 5 depicts the fundamental operations of standard convolution.

**Figure 5:** Convolution in the conventional sense.

Classic convolutional comprises of two steps: first, a depthwise convolution layer filters the input, and then a 1×1 (or pointwise) convolution operation integrates the filtered values to create innovative features.

In a typical convolutional layer with *X*_*in*_ input channels and *X*_*out*_ output channels, each output feature map is the sum of the *X*_*in*_ input feature maps twisted by the *X*_*in*_ corresponding kernel.

A standard convolution has the following weights:


(1) $$\begin{array}{l} \;W_{std}=C_{in}{\;\times \;K}_{w}\;\times \;K_{H}\times \;C_{out}\;\\ Wgt_{std}=X_{in}{\;\times \;K}_{w}\;\times \;K_{H}\times \;X_{out} \end{array}$$

The kernel size is denoted by the symbols *K*_*w*_ × *K*_*H*_.

Generating outcome feature maps of dimension *f*_*w*_ × *f*_*H*_ has a computational load of:


(2) $$\begin{array}{l} \text{CCos}{\text{t}}_{\text{std}}={\text{X}}_{\text{in}}\;\times \;{\text{K}}_{\text{w}}\;\times \;{\text{K}}_{\text{H}}\times \;{\text{X}}_{\text{out}}\;\times \;{\text{f}}_{\text{w}}\;\times \;{\text{f}}_{\text{H}} \end{array}$$

Where K_w_ and K_H_ are the spatial dimensions (height and width) of the kernels, X_in_ and X_out_ are the count of input and output streams, and f_w_ and f_H_ are the spatial measurements maps of the outcome.

#### Depthwise Separable Convolutional Neural Network Based on Mobile Net Architecture

In this section, we'll go over the depth-separable filters that form the foundation of MobileNet. The Depthwise Separable Convolutional Neural Network based on MobileNet is next described in detail. The MobileNet CNN (1) design is a form of the CNN model which can be used for developing deep neural networks in cellular systems. In terms of efficiency, it is a very effective way of building convolutional neural networks. One of the things that distinguishes it from other similar products is the use of Depthwise separable convolution.

***Depthwise and Pointwise Convolutions:*** The multi-layered features, as well as the contrast between conventional and depth-wise separable, are depicted in Figure 6. As illustrated in Figure 6, the Depthwise (dw) and pointwise (pw) convolutions are merged to create a “Depthwise separable” convoluted structure. The Depthwise separable convolutional structure provides a function comparable to traditional convolution but at a much faster rate. Because the frames are Depthwise separable, there's also no pooling layer between them in the given technique. A stride of two is included in a couple of the depth-wise layers to reduce spatial dimension. The collection of output channels is also included in the following pointwise layer in this case.

**Figure 6:** Depthwise separable convolution.

Figure 6 shows the fundamental methods of Depthwise convolution and Depthwise separable convolution. In contrast to conventional convolution, Depthwise convolution creates only one output feature space from a single input matrix modified by a single convolution operation (5).


(3) $$\begin{array}{l} \text{Wg}{\text{t}}_{\text{dws}}={\text{K}}_{\text{w}}\;\times \;{\text{K}}_{\text{H}}\times \;{\text{X}}_{\text{out}} \end{array}$$

The expense of computing a Depthwise convolution layer is as follows:


(4) $$\begin{array}{l} CCost_{dws}={\;K}_{w}\;\times \;K_{H}\times {\;X}_{in}\times {\;f}_{w}\times \;f_{H}\;+{X_{in\;}\times \;X}_{out}\\ \;\times \;{\;f}_{w}\;\times \;f_{H} \end{array}$$

Employing Depthwise convolution, the weighting and calculation cost are decreased by X_in_ times.

A DWS convolution is similar to a traditional convolution because it decreases the computational complexity by a proportion of α, which would be denoted by Equation (5).


(5) $$\begin{array}{l} \alpha =CCost_{reduced}=\frac{CCost_{dws}}{CCost_{std}} \end{array}$$

(6) $$\begin{array}{l} \alpha =\frac{K_{w}\times K_{H}\times X_{out}\times f_{w}\times f_{H}+{X_{in}\times X}_{out}\times f_{w}\times f_{H}}{X_{in}{\times K}_{w}\times K_{H}\times X_{out}\times f_{w}\times f_{H}} \end{array}$$

(7) $$\begin{array}{l} \alpha =\frac{1}{X_{in}}+\frac{1}{K_{w}\;\times \;K_{H}} \end{array}$$

The calculations can be further illustrated as follows:

The depth-wise separable convolution has two parts: depth-wise and point-wise convolution. It uses depth-wise convolution to apply a singular filtering on all transmissions of input vectors. The depth-wise convolution is expressed by Equation (8).


(8) $$\begin{array}{l} F\left(a,b,i\right)=\overset{m}{\underset{v=1}{\sum }}\overset{m}{\underset{v=1}{\sum }}M\left(v,v,i\right)\times \;N\left(a+v-1,\;v-1,i\right) \end{array}$$

wherein m represents depth-wise convolutional kernels of size m x m x cin and cin symbolizes convolutional kernels of dimension m x m x cin. The nth filter in M is deployed to the nth channel in N to create the nth channel of the filtration outcome feature vector F.

A point-wise convolution uses 1x1 convolution to determine the linearly separable clustering of the depth-wise convolution outcome for generating new features. A point-wise convolution is expressed by Equation (9).


(9) $$\begin{array}{l} P\left(a,b,j\right)=\overset{cin}{\underset{i=1}{\sum }}M\left(v,v,i\right)\times \;Q\left(i,j\right) \end{array}$$

The size of the 1x1 convolutional kernel is **1 × 1 ×** ***Xin*** **×** ***Xout***. Changing m changes the total number of channels in the output feature vector. The dense 1×1 convolutional function, like the m x m (m > 1) convolutional functions, has no requirement for being close to the vicinity, therefore changing the configuration in memory is not required. After then, the operation is carried out horizontally utilizing very efficient fundamental matrix multiplication algorithms. A DWS convolution computation is expressed by Equation (10):


(10) $$C_{\text{dws}\text{=}m^{2}\;.\;c_{in}\;.\;h.\;w+x_{in}.\;x_{out}.\;h\;.\;w\;}$$

It expresses the expense of convolution layer and 1x1 point-wise convolutional computations.

The connecting strengths in a Depthwise convolution are as follows: The percentage n is generally equivalent to 1/k2 since the magnitude of m is frequently rather big. Since this study employs 3×3 DWS convolution layers, the computational cost and parametric densities of comparable convolution operation are 7 to 8 times smaller than conventional convolution operation.

***How it Works***: In order to increase the real-time performance of the network learning under constrained hardware settings, the Depthwise Separable Convolutional Neural Network based on MobileNet (3) was designed. It's possible to minimize the number of parameters while still getting good results with this network. Depthwise Separable Convolutional Neural Network based on MobileNet's fundamental convolution structure is seen in Figure 7. Deep and severable convolution structure, Conv Dw Pw. For example, it has a depth-wise (Dw) and point-wise (Pw) structure (Pw). Three-layer convolutions are used in the Dw, whereas one-layer convolutions are used in the Pw. The batch normalization procedure as well as the activation function rectified liner unit (ReLU) are applied to each convolution result. The suggested Depthwise Separable Convolutional Neural Network based on MobileNet architecture is is built with Tensorflow and includes the depthwise convolution layer structure. It should be noted that after each convolution, Batch Normalization (BN) and ReLU are executed as follows (Figure 7).

**Figure 7:** Depth-wise: separable convolutions with depth-wise and pointwise layers, then batchnorm and ReLU, are the next steps.

On the basis of the Depthwise Separable Convolutional Neural Network based on MobileNet architecture, we designed this deep learning model with the goal of improving efficiency while being lightweight enough to be deployed on smartphones. This version of t uses depth-separable convolution as the basis for its efficient construction (23). Afterward, each layer has a batchnorm (10) and a ReLU non-linearity. The last fully connected layer has no non-linear behavior and enters into a softmax function for categorization. The number of layers in MobileNet is 28 if you consider Depthwise and pointwise convolutions to be different layers. The proposed structure places virtually all of the processing into dense 1x1 convolutions, which reduces the amount of computing required. This may be accomplished through the use of highly efficient generalized matrix multiplying routines.

***Implementation:*** We used Depthwise Separable Convolutional Neural Network based on MobileNet architecture, which is an effective method for lowering the computation complexity of deep learning models. It consists of a 1×1 convolution output node with spatial convolution performed independently on each pulse (24). We utilized the convolution layer's output as a feed to the Rectified Linear Unit (ReLU) activation function, with a 1-dimensional max pooled on the result. The filtering size and depth of the first convolutional layer are both adjusted to 60, whereas the pooling layer's filter size is fixed to 20 with a step number of 2.

For the fully linked layer input, the result of the succeeding convolution operation is flattened down to a stepping of six. After obtaining an intake from the max-pooling layer, the convolution layer employs a filter of various sizes, which has 10% of the max-pooling layer's complexity. For the completely connected layer input, the result is smoothed down. According to the aforementioned design, the completely associated layer comprises 1,001 neurons. The hyperbolic tangent function represents non-linearity in the current layer. To calculate the probability for the corresponding target tags, the Softmax function is utilized. To reduce the potential log-likelihood objective functions, the stochastic gradient descent optimizing approach was utilized. Each functional map's matrix description is converted to a vector via the flattening layer. Several dropouts are mounted on the top of the pooling layer to eliminate the potential for overfitting. The suggested system includes a max-pooling layer that sums the feature maps generated by the convolution layers and reduces computing costs. In order for the Depthwise Separable Convolution Neural Network (DS-CNN) to operate, the volume of the function mappings must always be reduced, along with their size. In the proposed model configuration, the final layer is a totally connected layer, accompanied by a Softmax classifier to efficiently classify facial images. Depth-separable convolutions are used in the suggested MobileNet method. The overall number of learnable parameters in our system is 6,844, as opposed to 14,362 for the very same system using traditional convolutions. We chose this particular DS-CNN because of its demonstrated versatility, training efficacy, low parameter bank, and impressive performance on smaller samples (25).

## Results and Discussion

This section summarizes and evaluates the information gathered by establishing experiment setups and conducting multiple trials to address the research questions.

### Answering Research Question No. 1

To get a solution to RQ1: **“***How can the Depthwise Separable Convolutional Neural Network based on MobileNet be utilized to successfully categorize photos for facial mask detection?*, we would examine at the hardware and the software which will be used to create the recommended system. The parameters for training and performance of the depth-wise separable convolutional network structure are therefore fully explored.

#### Hardware and Software Configuration

For the tests, we used an Intel Core i7 CPU, an Nvidia GTX 1080 GPU, and Windows 10. Python 3.5 was utilized as the programming language. It uses Python 3.5's PyTorch library and MATLAB 2019b for image embedding processing and analysis, respectively. 224 × 3 STIF frames are all that is needed to use the pre-trained model. This dataset is used to test the suggested method, which is detailed in section Answering Research Question No. 1 below. Training and testing datasets have been created. Initially, the scaling factor was set at 0.001, and it drops by a factor of 0.9 every 10 epochs after that. A momentum value of 0.999 is utilized in the Adam optimizer. Until 100 epochs have passed, the training procedure is repeated.

#### Parameter Setting

The design of the suggested MobileNet parameter settings for effective categorization of facial images (Mask/no-mask) is adopted from (23).

#### Implementation of Facial Image Classification in Terms of Mask/No-Mask

For the deployment of classification system for facial images, Table 3 shows the distribution of processor time for a particular deductive logic over network layers. With three interpretations per second, the network analysis took adequate time for feature extraction and image source processing.

**Table 3:** Layered process time distribution and classification assessment tasks.

**Layer**	**Execution time [% of ms]**	**Millions of operations (%)**
Conv1	41.01%	21.1%
DWS_Conv1	2.9%	0.08%
Pw_Conv1	3.5%	8.1%
DWS_Conv2	2.8%	0.02%
Pw_Conv2	3.3%	7.7%
Pooling_avg	0.2%	0.1%

### Responding to Research Question No. 2

To assess the proposed model for detecting mask detection in facial images, we tested the performance of Full Convolution MobileNet models on the obtained datasets to answer RQ2: “*How efficient is the suggested technique in contrast to the traditional CNN model in terms of many performance assessment measures?”*

#### Experimental Results

There is only a limited number of labeled samples. Therefore, decreasing the hyperparameters improves training. Hence, the convolution kernel's dimension in the neural network is set at 1×1. A final result of 5 × 5 × 64 is obtained by increasing the number of filters per layer to 64 at the same time. For the sake of reproducibility, the training photos for each experiment were randomly picked from a pool of facial photographs. As a result, the model's training efficiency and processing costs are both reduced by the compact Depthwise separable convolutional network model. The confusion matrix of the MobileNet (DWS-based) model in a laboratory environment may be shown in Figure 8.

**Figure 8:** Confusion matrix.

#### Contrast of the Suggested MobileNet (DWS-CNN-Based) With the Full Convolution MobileNet

Table 4 displays the computation cost as the total number of multipliers of one frame data in convolution-based layers for the forward run. The total number of learnable model parameters is also calculated. Table 4 compares the efficacy of the recommended technique, namely MobileNet (Depthwise separable convolutional network) to that of a Full Convolution MobileNet. It also indicates that, as compared to Full Convolution MobileNet, using Depthwise separable convolution-based CNN enhances accuracy by 0.6 percent while dramatically lowering computations times and trainable parameters. The results of the experiment and complexity analysis demonstrate that the proposed model may be used in spectral image-based applications with reasonable accuracy.

**Table 4:** DWS-based (MobileNet) (proposed) and full convolution MobileNet performance comparison.

	**Accuracy (avg. percent)**	**Overhead in computing (in min.)**	**Parameters**
Full convolution MobileNet	92.008	8.428	14, 362
MobileNet (DWS-based) (proposed)	93.164	2.106	6, 844

#### Cross Validation Results for Classification Techniques

The 10-fold cross-validation technique was used to test classification models. Table 5 displays the findings of the average accuracy, standard deviation (accuracy), precision Marco (average), standard deviation (precision Marco), recall Marco (avg.), standard deviation (recall Marco), average F-1 Marco, and standard deviation F-1 Marco. These factors will assist us in evaluating and forecasting the effectiveness of the proposed MobileNet (DWS-based) model for the classification of facial images. Table 5 shows that the greatest average accuracy in the AIZOO FACE MASKS dataset is 93.621 percent when compared to SVM and CNN.

**Table 5:** Cross validation results.

**Model**	**Avg. Accuracy**	**St. dev. (Acc.)**	**Avg. prec. macro**	**St. dev. (prec. Macro)**	**Avg. rec. macro**	**St. dev**.	**Avg. FI macro**	**St. dev**.
SVM	92.008	0.06	85	0.05	89	0.07	87	0.07
CNN	91.03	0.06	86	0.05	88	0.06	86	0.06
MobileNet (DWS-based)	93.164	0.05	90	0.04	91	0.05	89	0.05

Among the most frequently used classification methods for face image analysis, SVM and CNN are the most generally employed because of their effectiveness, performance, and ability to handle a large feature set with a large number of features. Classification challenges may be solved using these supervised learning approaches. Using the SVM (26), each element's relevance is represented as a score for a specific arrangement. Instead of attempting to categorize the two groups, locate the hyper-plane that best separates them.

Using the AIZOO FACE MASKS dataset, three approaches were used to create the classification maps in Figure 9.

**Figure 9:** Three techniques' classification maps using AIZOO FACE MASKS dataset. **(A)** MobileNet (DWS-based) (proposed), **(B)** Full Convolution MobileNet, and **(C)** CNN.

#### Evaluation of Performance

The effectiveness of the recommended model is examined using four evaluation metrics as follows (26–29):

(i) ***Accuracy:***
  We quantify classification accuracy using Equation (11) to highlight the usefulness and reliability of the suggested method.
  (11) $$\begin{array}{l} Accuracy=\frac{TP+TN}{TP+TN+FN+FP}\\ \;TP=\text{true positive},\;TN=\text{true negative},FP=false\\ \;positive,and\;FN=\text{false negative} \end{array}$$
(ii) ***Precision:***
  Precision is a positive prediction number that shows how correct the system is. For a limited number of false-positive criteria, precision rises substantially. The following is a mathematical equation to consider.
  (12) $$\begin{array}{l} Precision\left(p\right)=\frac{TP}{FP+TP}\\ \;p=precision,\;TP=\text{true positive},\;FP=false\\ \;positive,and\;FN=\text{false negative} \end{array}$$
(iii) ***Recall:***
  It's also referred to as sensitivity, and it indicates how many confident instances the model properly identifies. When the recall is large, the proportion of +ive cases incorrectly classified as –ive is smaller. A mathematical expression is as follows:
  (13) $$\begin{array}{l} Recall\left(r\right)=\frac{TP}{FN+TP}\\ \;r=recall,TP=\text{true positive},\;and\\ \;FN=\text{false negative} \end{array}$$
(iv) ***F-measure:***
  The mean of recall and precision is the F-score or F1-Measure. The following is a mathematical formula for calculating it:
  (14) $$\begin{array}{l} F_{measure}=\frac{TP}{TP+\frac{1}{2}\left(FP+FN\right)}\\ \;R=Recall,P=Precision,TP=\text{true positive},\\ \;FP=\text{false positive},\;and\;FN=\text{false negative} \end{array}$$

Based on Face Mask Detection Using MobileNet's precision and recall statistics, we can learn more about our model's performance.

That the model can accurately identify face photos (mask or no mask) with promising precision and recall is demonstrated in Table 6 (sensitivity). As a result of the model's strong recall and precision findings in the experiment, it has a great deal of promise for minimizing the number of false positives and negatives in facial mask detection applications during the COVID-19 pandemic. For real-time face photos, the model's average classification time of 1,020 samples was 2.5 s, making it suitable for mask and no-mask classification.

**Table 6:** DWS (based on MobileNet) results for facial image (mask/no mask) classification.

**Mask/No-Mask Class**	**Precision (%)**	**Recall (%)**	**F-score (%)**
Mask	96	96	95
No-Mask	97	96	97

### Answering the Third Research Question

While answering RQ3: “*What is the effectiveness of the suggested approach in comparison to comparable approaches?”*, we evaluated the effectiveness of the baseline on the given dataset to assess the proposed Depthwise Separable-based MobileNet model for hyperspectral images. We also conducted a statistical assessment to verify the usefulness of the proposed technique.

#### Using the Base Line Methods as a Point of Reference for Comparison

On the same dataset, we employed the 10-fold cross validation method to compare our system to the previous facial mask classification research published in (2). Deep CNN classification algorithms were also used to construct a system for analyzing data. Table 7 shows the comparison between precision and the F1 measure in terms of precision. Compared to the baseline framework, the suggested model has a higher sensitivity and an F1-score. There has been a noticeable increase in the suggested platform's capacity to recognize and remember classifications of face pictures in the mask detection scenario.

**Table 7:** Comparative results to benchmark work.

**Mask/No-mask class**	**Kaur et al**. **(****2****)**			**Fan et al**. **(****3****)**			**Proposed framework**		
	***P* (%)**	***R* (%)**	**F1 (%)**	***P* (%)**	***R* (%)**	**F1 (%)**	***P* (%)**	***R* (%)**	**F1 (%)**
Mask	88	90	89	90	91	91	95	93	94
N-Mask	90	89	89	91	90	90	93	92	92

## Conclusion and Future Work

This study proposes the MobileNet-based Depthwise Separable Convolution Neural Network (DS-CNN) for mask detection in facial images. We compare our findings to the original convolutional filters on specific datasets. The suggested system outperformed current classical convolutions in experiments, according to the results. The suggested technique is also contrasted with previous work on a motivated baseline method. Our findings (Acc. = 93.14, Pre. = 92, recall = 92, F-score = 92) show that the proposed method produces the highest overall performance across a variety of assessment metrics. The approach requires extra processing to generate visualizations and, owing to dataset constraints, cannot discriminate between right and erroneous mask usage. Our future aim is to create face mask recognition datasets with different mask wearing states, or employ zero shot learning to make the design identify erroneous mask wearing states.

## Data Availability Statement

The raw data supporting the conclusions of this article will be made available by the authors, without undue reservation.

## Author Contributions

All authors listed have made a substantial, direct, and intellectual contribution to the work and approved it for publication.

## Funding

The APC was funded by Taif University Researchers Supporting Project Number (TURSP-2020/331), Taif University, Taif, Saudi Arabia.

## Conflict of Interest

The authors declare that the research was conducted in the absence of any commercial or financial relationships that could be construed as a potential conflict of interest. The handling editor declared a past co-authorship with one of the authors JA.

## Publisher's Note

All claims expressed in this article are solely those of the authors and do not necessarily represent those of their affiliated organizations, or those of the publisher, the editors and the reviewers. Any product that may be evaluated in this article, or claim that may be made by its manufacturer, is not guaranteed or endorsed by the publisher.
